The article "Knockdown of circRNA_0007534 suppresses the tumorigenesis of cervical cancer via miR-206/GREM1 axis" was retracted in 2022. Reasons: duplicated images; original data or images not available; unreliable data.

# Knockdown of circRNA_0007534 suppresses the tumorigenesis of cervical cancer via miR-206/GREM1 axis

**DOI:** 10.1186/s12935-021-01749-7

**Published:** 2021-01-14

**Authors:** Qiang Sun, Xiangying Qi, Wenyan Zhang, Xiaoyu Li

**Affiliations:** 1 Department of Obstetrics and Gynecology, Zaozhuang Municipal Hospital, No. 41, Longtou Road, Zaozhuang, 277100 Shandong China; 2 Department of Pharmacology, Shandong Academy of Chinese Medicine, Jinan, Shandong China

**Keywords:** Circ_0007534, Cervical cancer, miR-206, GREM1

## Abstract

**Background:**

Increasing evidence manifested that circular RNAs (circRNAs) acted as crucial regulators in human cancers by targeting the miRNA/mRNA axis, including cervical cancer (CC). Circ_0007534 was reported to promote CC cell proliferation and invasion by the miR-498/BMI-1 axis. The aim of this study was to explore a novel miRNA/mRNA network underlying circ_0007534 in CC regulation.

**Methods:**

The quantitative real-time polymerase chain reaction (qRT-PCR) was implemented to examine the levels of circ_0007534, miR-206 and Gremlin1 (GREM1). Cell viability was determined using MTT assay. BrdU and colony formation assays were performed for analyzing cell proliferation. Cell apoptosis was assessed by flow cytometry. The protein levels of GREM1 and apoptotic markers (Bcl-2, Bax, C-Caspase3) were measured via western blot. Cell invasion was detected by transwell assay. The target relationship was analyzed by dual-luciferase reporter assay. The impact of circ_0007534 on CC growth in vivo was ascertained by xenograft assay.

**Results:**

Circ_0007534 expression was aberrantly increased in CC tissues and cells. Functionally, knockdown of circ_0007534 reduced CC cell growth and invasion but motivated apoptosis. In the mechanism, circ_0007534 targeted miR-206 and its regulatory function was associated with sponging miR-206. Moreover, circ_0007534 was found to regulate GREM1 level by targeting miR-206. The inhibitory effect of si-circ_0007534 on the malignant progression of CC was reversed after GREM1 was overexpressed. Furthermore, circ_0007534 inhibition also reduced tumor growth of CC in vivo partially by regulating miR-206/GREM1 axis.

**Conclusion:**

These results suggested that knockdown of circ_0007534 promoted the level of miR-206 to induce the expression downregulation of GREM1, consequently inhibiting the progression of CC.

## Highlights

1. Circ_0007534 is expressed at a high level in CC tissues and cells.
2. Knockdown of circ_0007534 reduces proliferation and invasion while motivates apoptosis in CC cells.
3. Down-regulation of circ_0007534 refrains GREM1 expression by promoting miR-206.
4. Inhibition of circ_0007534 inhibits tumor growth partly by miR-206/GREM1 axis.

## Introduction

Cervical cancer (CC) is a gynecological malignancy accounting for a considerable proportion of cancer-associated death in females [1]. The risk factors for CC include human papilloma virus (HPV) infection, tobacco smoke and multiple sexual partners [2]. Modern treatment of CC has been developed and HPV vaccination is the most effective means to prevent CC [3]. CC is relatively rare in high-income countries because of the organized vaccination inoculation [4]. 90% of deaths from CC are found in low- and middle-income countries (especially in the areas of high HIV prevalence) due to the scarcity of preventive opportunity and limitation of treatments [5]. The recent research has reported that CC burden has been increased in southern Africa and eastern Africa [6]. To seek therapeutic targets and explore the pathological mechanism may be beneficial for the diagnosis and treatment of CC patients.

Circular RNAs (circRNAs) are known as the covalent closed-loop structures with the absence of 3′ tails and 5′ caps, and they have high stability to resist the external degradation [7, 8]. CircRNAs have regulatory effects on tumorigenesis and tumor progression by acting as the sponges of microRNAs (miRNAs) to regulate the gene expression [9, 10]. In CC, circRNA_0023404 has been proved to serve as an oncogenic regulator by affecting the miR-136/YAP axis [11] and circHIPK3 promoted the progression of CC via modulating the miR-485-3p/FGF2 axis [12]. In addition, the circ_0007364/miR-101-5p/MAT2A axis and circ_0084927/miR-634/TPD52 axis were also found in the development of CC [13, 14]. Circ_0007534 is derived from DEAD box polypeptide 42 (DDX42) gene in the chr17: 61869771-61877977, and it has been identified as a carcinogene in many types of cancers [15–17]. Rong et al. showed that circ_0007534 accelerated the proliferation and invasion of CC cells via the miR-498/BMI-1 axis [18]. Nevertheless, the other molecular mechanism of circ_0007534 in CC is unclear.

MicroRNA-206 (miR-206) is a common anti-cancer molecule. CircRNA cZNF292 and circ_0056618 have been respectively proved to promote the cancer progression in esophageal cancer and gastric cancer by targeting miR-206 [19, 20]. MiR-206 was shown to reduce cell growth and metastasis in CC cells [21]. However, it remains unreported whether miR-206 can be a target of circRNA (such as circ_0007534) in CC. MiRNAs can combine with the 3′-untranslated regions (3′-UTRs) to affect the expression of downstream target in cancer regulation [22]. The previous studies have revealed that miR-206 suppressed CC proliferation and invasion by targeting BAG3 and G6PD [23, 24]. Gremlin1 (GREM1), the subfamily of bone morphogenic protein (BMP) antagonists, has crucial regulation on body formation, skeleton patterning and organogenesis [25]. GREM1 expression was upregulated in diverse kinds of cancers, including CC [26]. It is also unexplicit about the potential of GREM1 as a downstream target of miR-206 in CC.

Herein, we assumed that miR-206 was a target of circ_0007534 and GREM1 was a target gene of miR-206. The influence of circ_0007534 on the GREM1 expression by targeting miR-206 was also explored in this study. Our research focused on the different molecular mechanism of circ_0007534 in regulating the developing process of CC.

## Materials and methods

### Tissues acquisition and cell culture

The present study was approved by the Ethics Committee of Zaozhuang Municipal Hospital. 35 pairs of CC tissues and normal contiguous tissues were collected from patients with CC at Zaozhuang Municipal Hospital. These patients have signed the written informed consent forms before the cervicectomy. The information of patients was shown in Table 1. All these tissues were rapidly stored in − 80 °C ultra-low temperature freezer (Thermo Fisher Scientific, Waltham, MA, USA).

**Table 1:** Correlation between circ_0007534 expression and clinical clinicopathological parameters of cervical cancer

Parameter	Case	Circ_0007534 expression		*P* value^a^
		Low (n = 17)	High (n = 18)	
Age (years)				0.130
≤ 60	16	10	6	
> 60	19	7	12	
Tumor size				0.001*
≤5 cm	15	12	3	
>5 cm	20	5	15	
TNM stages				0.004*
I–II	18	13	5	
III	17	4	13	
Vascular invasion				0.601
Absent	19	10	9	
Present	16	7	9	
Distant metastasis				0.024*
M_0_	12	9	3	
M_1_	23	8	15	

*TNM* tumor-node-metas-tasis; *P < 0.05, ^a^Chi square test

Human normal cervical cell line (Ect1/E6E7) and CC cell lines (Caski, C33A, SiHa and HeLa) were acquired from American Type Culture Collection (ATCC, Manassas, VA, USA). Cells were cultured in Dulbecco’s modified Eagle medium (DMEM; Gibco, Carlsbad, CA, USA) supplemented with 10% fetal bovine serum (FBS; Gibco) and antibiotics (100 U/mL penicillin and 100 μg/mL streptomycin; Gibco) in humidified air with constant conditions of 37 °C and 5% CO_2_.

### Cell transfection

Small interfering RNA (siRNA) against circ_0007534 (si-circ_0007534), miR-206 mimic (miR-206), miR-206 inhibitor (anti-miR-206) and the relative negative control (si-NC, miR-NC and anti-miR-NC) were purchased from GENEWIZ (Suzhou, China). Overexpression vectors of circ_0007534 and GREM1 were respectively constructed by inserting the sequence into the pCD5-ciR (GENESEED, Guangzhou, China) and pcDNA3.1 vector (Invitrogen, Carlsbad, CA, USA). Cell transfection was conducted using Lipofectamine3000 reagent kit (Invitrogen; L3000075). 1 × 10^4^ SiHa and HeLa cells were inoculated into the 96-well plates, then cultured to 70% monolayer confluence. Oligonucleotides/vectors were respectively diluted in Opti-MEM™ medium (Gibco), and added into the diluted Lipofectamine3000 reagent for 15 min. Subsequently, the mixture was pipetted into each well and cells were incubated at 37 °C to be used for the further analysis.

### Quantitative real-time polymerase chain reaction (qRT-PCR)

Total RNA was extracted by Trizol reagent (Invitrogen; 15596018) following the user’s manual. 2 μg RNA was reversely transcribed into the complementary DNA (cDNA) using PrimeScript™ RT Master Mix (Takara, Dalian, China; RR036Q) or Mir-X miRNA First-Strand Synthesis Kit (Takara; 638315). The qRT-PCR was performed by TB Green^®^ Premix Ex Taq™ II Kit (Takara; RR82LR) and Mir-X miRNA qRT-PCR TB Green^®^ Kit (Takara; 638314). The calculation of the relative expression was performed using 2^−∆∆Ct^ method [27]. Glyceraldehyde-3-phosphate dehydrogenase (GAPDH; for circ_0007534, DDX42 and GREM1) and small nuclear RNA U6 (for miR-206) were used as the internal references. The primer sequences were listed in Table 2.

**Table 2:** Primer sequences used for qRT-PCR

Name	Primer sequences
Circ_0007534	Forward: 5′-CTGGTGTGGTTCAGGAGGAA-3′
	Reverse: 5′-ATGGAATTGCTGGCGAGTTG-3′
DDX42	Forward: 5′-CCGCTCGAGAGGGGATGTGCTAAAGCGT-3′
	Reverse: 5′-GAATGCGGCCGCCCCGGTAGTAAAACATTTACTA-3′
miR-206	Forward: 5′-CCGGAATTCATGGT-3′
	Reverse: 5′-CCGATCGATTTAACTTTT-3′
GREM1	Forward: 5′-TAACACTGCCACAAGAATGCAA-3′
	Reverse: 5′-GCAAGACTGTGGTACAAGCTCCTAA-3′
GAPDH	Forward: 5′-TTGCCCTCAACGACCACTTT-3′
	Reverse: 5′-TGGTCCAGGGGTCTTACTCC-3′
U6	Forward: 5′-ATTGGAACGATACAGAGAAGATT-3′
	Reverse: 5′-GGAACGCTTCACGAATTTG-3′

### Ribonuclease R (RNase R) treatment

To measure the stability of circ_0007534, 2 μg total RNA was treated with 3 U/μg RNase R (Epicentre Technologies, Madison, WI, USA) at 37 °C. 30 min later, the expression levels of circ_0007534 and linear DDX42 were detected using qRT-PCR.

### MTT assay

MTT assay was used for cell viability analysis by CyQUANT™ MTT Cell Viability Assay Kit (Invitrogen, V13154). 1 × 10^4^ SiHa and HeLa cells were respectively seeded into the 96-well plates overnight. 10 μL MTT solution was incubated to cells after transfection for 0 h, 24 h, 48 h and 72 h. 4 h later, 100 μL dimethyl sulfoxide (DMSO; Invitrogen) was added to dissolve the formazan. The optical density (OD) value of 490 nm was read under the microplate reader (Thermo Fisher Scientific).

### BrdU assay

2 × 10^5^ cells were inoculated into a 6-well culture plate (with a cover slip placed inside) for 24 h, then incubated with 1.0 mg/mL BrdU solution (Applied Biosystems, Foster City, CA, USA) for 4 h. The culture solution was then discarded, followed by cell fixation in methanol for 10 min and cell staining in diamidine phenyl indoles (DAPI; Thermo Fisher Scientific). BrdU-positive cells were arbitrarily counted in three visual fields through the microscope.

### Colony formation assay

SiHa and HeLa cells (at 72 h post-transfection) were plated into the 6-well plates at the density of 200 cells/well. Cell culture was performed for 2 weeks until the macroscopic white colonies were emerged. Then cells were fixed using methanol and dyed with Giemsa (Sigma-Aldrich, St. Louis, MO, USA). The number of colony (more than 50 cells as one colony) was counted under the microscope.

### Flow cytometry

SiHa and HeLa cells (1 × 10^4^ cells/well) were seeded into the 96-well plates, then 3 × 10^4^ cells were collected using trypsin (Gibco) after transfection for 48 h. Whereafter, cells were doubly stained by Annexin V-fluorescein isothiocyanate (Annexin V-FITC) and propidium iodide (PI) using Annexin V-FITC Apoptosis Detection Kit (Sigma-Aldrich; APOAF-50TST) according to the manufacturer’s instruction. The apoptotic cells were discerned by the flow cytometer (Becton–Dickinson, San Jose, CA, USA).

### Western blot

Total proteins were lysed using RIPA lysis buffer (Sigma-Aldrich) and separated by sodium dodecyl sulfate–polyacrylamide gel electrophoresis (SDS-PAGE). After the proteins were transferred to polyvinylidene fluoride (PVDF) membranes (Abcam, Cambridge, United Kingdom), the non-specific protein binding was blocked by immersing the membranes in 5% skim milk (Thermo Fisher Scientific) for 3 h. Then the membranes were incubated with anti-B cell lymphoma-2 (anti-Bcl-2; Abcam, ab32124, 1:1000), anti-Bcl-2-Associated X (anti-Bax; Abcam, ab32503, 1:1000), anti-Cleaved-Caspase3 (anti-C-Caspase3; Abcam, ab32503, 1:1000), anti-GREM1 (Abcam, ab140010, 1:1000) and anti-GAPDH (Abcam, ab9485, 1:3000) at 4 °C overnight. PVDF membranes were washed using 0.05% PBS with Tween 20 (PBST; Invitrogen), followed by the incubation of the secondary antibody (Abcam, ab205718, 1:5000) at room temperature for 45 min. Ultimately, the protein bands were detected using the enhanced chemiluminescence reagent (Sigma-Aldrich) and the protein expression was analyzed under the Image J software (NIH, Bethesda, MD, USA).

### Transwell invasion assay

The upper chamber of transwell 24-well chamber (Corning Life Sciences, Corning, NY, USA) was coated with matrigel (Corning Life Sciences), then seeded with 1 × 10^4^ SiHa or HeLa cells. The lower chamber was added with fresh 600 µL DMEM medium containing 10% FBS. After incubation for 24 h, cells were fastened and stained using methanol and crystal violet (Sigma-Aldrich). The invaded cells from the upper chamber into the lower chamber were counted under an inverted microscope (Olympus, Tokyo, Japan). Cell images were acquired at the 100 × magnification.

### Dual-luciferase reporter assay

Starbase was used for the target prediction of circ_0007534 and miR-206. The sequences of circ_0007534 and 3′UTR of GREM1 containing the binding sites of miR-206 were inserted into the pmirGLO basic vector (Promega, Madison, WI, USA), then the wild-type (WT) luciferase reporter plasmids were named as circ_0007534 WT and GREM1 3′UTR WT. After the binding sites were mutated, the mutant-type (MUT) luciferase plasmids (circ_0007534 MUT and GREM1 3′UTR MUT) were constructed as the above description. SiHa and HeLa cells were transplanted into the 48-well plate with 3 × 10^4^ cells per well, then 2 µL plasmid was co-transfected with 100 nM miR-206 mimic or miR-NC into the monolayer cells. Cells were harvested after transfection for 48 h and lysed in 1 × Passive Lysis Buffer (Promega). The supernatants were transferred into a new tube after the centrifugation for 10 min at 12,000 rpm, then the firefly and renilla luciferase activities were detected using the dual-luciferase reporter system (Promega; E1910). The ratio of firefly and renilla activity was considered as the relative luciferase activity.

### Establishment of stably transfected cells

Lentivirus vectors of short hairpin RNA (shRNA) against circ_0007534 (sh-circ_0007534) and negative control (sh-NC) were bought from RIBOBIO (Guangzhou, China). HeLa cells in logarithmic growth phase were seeded on the 24-well plates with the initial cell density of 5 × 10^4^/well. After 24 h, HeLa cells were injected with lentiviruses with the best multiplicity of infection (MOI = 20) that was explored in the pre-experiments. Cell medium was changed after 8 h and the stable cell lines with knockdown of circ_0007534 were acquired through the limited dilution method after the screening with antibiotic.

### Xenograft tumor assay

Six-week-old BALB/c female nude mice (n = 10) were bought from Vital River Laboratory Animal Technology Co., Ltd. (Beijing, China) and divided into two groups with 5 mice per group. Mice were cared in specific pathogen-free (SPF) environment with a constant temperature of 26 °C, a humidity of 70% and a programmed cycle of 12-h light/dark. Mice were subcutaneously injected with the established stable HeLa cells of sh-circ_0007534 or sh-NC, respectively. Tumors in mice were monitored every 5 days after cell injection. The length and width of tumors were measured using a digital caliper, followed by the calculation of tumor volume through the formula: (length × width^2^)/2. After the 25 d-observation, mice were euthanatized by displacing the 60% air of cage using the flow rate of CO_2_ in compliance with the current guideline of American Veterinary Medical Association (AVMA). Then tumors were excised from mice and weighed on an electronic scale, and the expression detection (for circ_0007534, miR-206 and GREM1) was performed using qRT-PCR or western blot. This animal experiment was ratified by the Experimental Animal Ethics Committee of Zaozhuang Municipal Hospital. All animal operations were performed following the guidelines of Animal Care and Use Committee of the National Institutes of Health.

### Statistical analysis

The biostatistical analysis was carried out using SPSS 19.0 and GraphPad Prism 7. The assays in this study were independently conducted for three times with three technical replicates. Data were presented as the mean ± standard deviation (SD). The difference analysis was performed by Student’s *t*-test or one-way analysis of variance followed by Tukey’s test. Statistically, the difference was identified as significant if *P *< 0.05.

## Results

### Circ_0007534 was highly expressed in CC tissues and cells

The qRT-PCR was performed to detect the level of circ_0007534 in CC tissues and cells. Results manifested that the expression of circ_0007534 was evidently increased in CC tissues (Fig. 1a) and CC cell lines (Caski, C33A, SiHa and HeLa) (Fig. 1b), in comparison with the normal tissues and Ect1/E6E7 cell line. SiHa and HeLa cell lines with more significant upregulation of circ_0007534 were chosen for the subsequent research in vitro. To evaluate the stability of circ_0007534, total RNA from SiHa and HeLa cells was treated with RNase R. The data of qRT-PCR showed that circ_0007534 was more resistant to RNase R degradation than linear DDX42 in SiHa (Fig. 1c) and HeLa (Fig. 1d) cells. Therefore, circ_0007534 was identified as a circRNA and its expression was upregulated in CC.

**Fig. 1:** Circ_0007534 was highly expressed in CC tissues and cells. **a**, **b** The qRT-PCR was conducted to examine the significant upregulation of circ_0007534 expression in CC tissues compared to healthy tissues (**a**) and CC cell lines compared to normal cervical epithelial cell line (**b**). **c**, **d** The qRT-PCR after RNase R treatment affirmed that circ_0007534 was more stable than linear DDX42 in SiHa (**c**) and HeLa (**d**) cells. CC: cervical cancer, DDX42: DEAD box polypeptide 42. All assays were performed for three times with technical n = 3. Statistical analysis was conducted by Student’s t-test and one-way analysis of variance followed by Tukey’s test. *P < 0.05, **P < 0.01, ***P < 0.001

### Down-regulation of circ_0007534 repressed CC cell growth and invasion but facilitated apoptosis

To explore the biological role of circ_0007534 in CC, SiHa and HeLa cells were respectively transfected with si-circ_0007534 and si-NC. The qRT-PCR result indicated that circ_0007534 expression in si-circ_0007534 group was much lower than that in si-NC group (Fig. 2a), implying that si-circ_0007534 successfully interfered the expression of circ_0007534. Subsequently, MTT assay revealed that transfection of si-circ_0007534 inhibited cell viability contrasted to si-NC transfection (Fig. 2b, c). Colony formation ability was also reduced in SiHa and HeLa cells transfected with si-circ_0007534 (Fig. 2d, e). BrdU assay exhibited the repressive effect of si-circ_0007534 (relative to si-NC) on proliferation of SiHa and HeLa cells (Additional file 1: Fig. S1). Flow cytometry demonstrated that the apoptotic rate of si-circ_0007534 group was higher than that of si-NC group (Fig. 2f, g). Western blot was used to analyze the levels of apoptosis-related makers. As depicted in Fig. 2h, i, the expression inhibition of circ_0007534 evoked the downregulation of Bcl-2 (anti-apoptotic protein) and the upregulation of Bax, C-Caspase3 (pro-apoptotic proteins). Moreover, transwell assay demonstrated that the invasive cell number was decreased after circ_0007534 knockdown (Fig. 2j, k). These results suggested that CC cell progression was impeded by the down-regulation of circ_0007534.

**Fig. 2:** Down-regulation of circ_0007534 repressed CC cell growth and invasion but facilitated apoptosis. **a** The qRT-PCR indicated that the interference efficiency of si-circ_0007534 was successful. **b**, **c** MTT displayed that si-circ_0007534 suppressed cell viability in SiHa (**b**) and HeLa (**c**) cells contrasted to si-NC. **d**, **e** Colony formation assay exhibited that si-circ_0007534 reduced cell proliferation contrasted to si-NC. **f**, **g** Flow cytometry demonstrated that si-circ_0007534 enhanced cell apoptosis contrasted to si-NC. **h**, **i** Western blot for apoptotic protein detection confirmed that cell apoptosis was promoted by si-circ_0007534 compared with si-NC. **j**, **k** Transwell assay suggested that cell invasion was inhibited by si-circ_0007534 compared with si-NC. *NC* negative control, *OD* optical density, *Bcl-2* B-cell lymphoma-2, *Bax* Bcl-2-Associated X, *C-Caspase3* Cleaved-Caspase3, *GAPDH* glyceraldehyde-phosphate dehydrogenase. All assays were performed for three times with technical n = 3. Statistical analysis was conducted by Student’s t-test. *P < 0.05, **P < 0.01, ***P < 0.001

### Circ_0007534 targeted miR-206 in CC cells

Starbase was applied for predicting the miRNA target of circ_0007534. As shown in Fig. 3a, the binding sites of miR-206 were found in circ_0007534. Dual-luciferase reporter assay manifested that the luciferase activity of circ_0007534 WT group was apparently reduced by miR-206 in SiHa and HeLa cells, while this inhibition was not observed in circ_0007534 MUT group (Fig. 3b, c). Compared to normal tissues and cells, miR-206 level was lower in CC tissues (Fig. 3d) and SiHa/HeLa cells (Fig. 3e). The downregulation of circ_0007534 induced the stimulative effect on the miR-206 expression in SiHa and HeLa cells (Fig. 3f). These data indicated that miR-206 was a target of circ_0007534.

**Fig. 3:** Circ_0007534 targeted miR-206 in CC cells. **a** Starbase showed the binding sites between circ_0007534 and miR-206. **b**, **c** The interaction between circ_0007534 and miR-206 was confirmed by dual-luciferase reporter assay in SiHa (**b**) and HeLa (**c**) cells. **d**, **e** The qRT-PCR identified the downregulation of miR-206 expression in CC tissues **d** by comparison with normal tissues and CC cells (**e**) by comparison with normal cells. **f** The qRT-PCR indicated that miR-206 level was elevated after knockdown of circ_0007534. *WT* wild-type, *MUT* mutant-type, *CC* cervical cancer, *NC* negative control. All assays were performed for three times with technical n = 3. Statistical analysis was conducted by Student’s t-test and one-way analysis of variance followed by Tukey’s test. *P < 0.05, **P < 0.01

### Overexpression of circ_0007534 relieved the miR-206-induced effects on CC cells by acting as a sponge of miR-206

The regulatory mechanism between circ_0007534 and miR-206 in CC was researched by the reverted transfection in SiHa and HeLa cells. By performing the qRT-PCR assay, we found that overexpression of circ_0007534 overtly prevented the up-regulation of miR-206 caused by miR-206 transfection (Fig. 4a). Transfection of circ_0007534 eliminated the suppressive effects of miR-206 on cell viability (Fig. 4b, c) and colony formation (Fig. 4d), as well as the stimulative effect on cell apoptotic rate (Fig. 4e). The introduction of miR-206 inhibited the protein level of Bcl-2 but upregulated the levels of Bax and C-Caspase3, whereas these effects were abrogated by circ_0007534 upregulation (Fig. 4f, g). Similarly, circ_0007534 mitigated the inhibition of cell invasion caused by miR-206 in SiHa and HeLa cells (Fig. 4h). Taken together, the function of circ_0007534 in CC progression was related to sponging miR-206.

**Fig. 4:** Overexpression of circ_0007534 relieved the miR-206-induced effects on CC cells by acting as a sponge of miR-206. **a** The qRT-PCR demonstrated that the miR-206-mediated high miR-206 expression was inhibited by circ_0007534 in SiHa and HeLa cells. (**b-d**) MTT and colony formation assay proved that circ_0007534 promoted cell viability (**b**, **c**) and proliferation (**d**) by upregulating the expression of miR-206. (**e–g**) Flow cytometry (**e**) and western blot (**f, g**) were performed to verify the regulation of circ_0007534/miR-206 axis in cell apoptosis. **h** Transwell assay validated that circ_0007534 facilitated cell invasive ability by targeting miR-206. *NC* negative control, *OD* optical density, *Bcl-2* B-cell lymphoma-2, *Bax* Bcl-2-Associated X, *C-Caspase3* Cleaved-Caspase3, *GAPDH* glyceraldehyde-phosphate dehydrogenase. All assays were performed for three times with technical n = 3. Statistical analysis was conducted by Student’s t-test and one-way analysis of variance followed by Tukey’s test. *P < 0.05, **P < 0.01, ***P < 0.001

### Knockdown of circ_0007534 repressed the GREM1 expression via upregulating miR-206

Target prediction of miR-206 was performed using Starbase, and the 3′UTR of GREM1 was found to have the binding sites of miR-206 (Fig. 5a). The luciferase activities of SiHa and HeLa cells co-transfected with GREM1 3′UTR WT and miR-206 were found to be suppressed, but no difference was noticed in luciferase activity after co-transfection of GREM1 3′UTR MUT and miR-206 (Fig. 5b, c). Through the analysis of qRT-PCR and western blot, we confirmed that GREM1 expression was upregulated in CC tissues (Fig. 5d, e) and SiHa/HeLa cells (Fig. 5f, g). Additionally, the GREM1 mRNA (Fig. 5h) and protein (Fig. 5i, j) levels were decreased by miR-206 in SiHa and HeLa cells. More interestingly, si-circ_0007534 led to the significant repression of GREM1 mRNA (Fig. 5k) and protein (Fig. 5l, m) expression while this influence was abrogated by miR-206 inhibitor. These findings proved that circ_0007534 could regulate the GREM1 expression via targeting miR-206.

**Fig. 5:** Knockdown of circ_0007534 repressed the GREM1 expression via upregulating miR-206. **a** The binding sites between miR-206 and GREM1 were presented by Starbase. **b, c** Dual-luciferase reporter assay exhibited the combination between of miR-206 and GREM1. **d-g** The qRT-PCR and western blot were conducted to determine the overexpression of GREM1 mRNA and protein levels in CC samples (**d, e**) relative to normal samples and CC cells (**f, g**) relative to normal cells. **h-j** The mRNA (**h**) and protein (**i, j**) levels of GREM1 were promoted by miR-206 mimic after the detection of qRT-PCR and western blot. (**k-m**) The si-circ_0007534-induced inhibitory effects on GREM1 mRNA (**k**) and protein (**l, m**) levels were restored by miR-206 inhibitor. *WT* wild-type, *MUT* mutant-type, *CC* cervical cancer, *GREM1* Gremlin1, *GAPDH* glyceraldehyde-phosphate dehydrogenase, *NC* negative control. All assays were performed for three times with technical n = 3. Statistical analysis was conducted by Student’s t-test and one-way analysis of variance followed by Tukey’s test. *P < 0.05, **P < 0.01

### Up-regulation of GREM1 reverted the effects of si-circ_0007534 on CC cells

The regulatory relation of circ_0007534 and GREM1 was further investigated in CC cells. GREM1 transfection lightened the si-circ_0007534-induced inhibitory effects on GREM1 mRNA (Fig. 6a) and protein (Fig. 6b, c) levels, showing that the overexpression efficiency of GREM1 vector was great. Subsequent functional experiments suggested that the inhibition of si-circ_0007534 on cell viability (Fig. 6d, e) and colony formation (Fig. 6f) but the promotion on cell apoptotic rate (Fig. 6g) and the changes on apoptotic proteins (Fig. 6h, i) were all counterbalanced by GREM1 overexpression. GREM1 transfection also restored the repression of si-circ_0007534 in cell invasion of SiHa and HeLa cells (Fig. 6j). Briefly, the effects of si-circ_0007534 on CC cells were all returned by overexpression of GREM1.

**Fig. 6:** Up-regulation of GREM1 reverted the effects of si-circ_0007534 on CC cells. **a-c** GREM1 transfection was shown to relieve the expression downregulation of GREM1 mRNA in qRT-PCR (**a**) and protein (**b, c**) in western blot caused by si-circ_0007534. **d-f** Cell viability inhibition in MTT (**d, e**) and proliferation repression in colony formation assay (**f**) by si-circ_0007534 were mitigated after transfection of GREM1. **g-i** The promotion of si-circ_0007534 on cell apoptosis was returned by the introduction of GREM1 through the analysis of flow cytometry (**g**) and western blot (**h**, **i**). **j** GREM1 transfection abolished the inhibition of cell invasion caused by si-circ_0007534 after performing transwell assay. *NC* negative control, *GREM1* Gremlin1, *OD* optical density, *Bcl-2* B-cell lymphoma-2, *Bax* Bcl-2-Associated X, *C-Caspase3* Cleaved-Caspase3, *GAPDH* glyceraldehyde-phosphate dehydrogenase. All assays were performed for three times with technical n = 3. Statistical analysis was conducted by Student’s t-test and one-way analysis of variance followed by Tukey’s test. *P < 0.05, **P < 0.01, ***P < 0.001

### Inhibition of circ_0007534 reduced tumor growth partly by increasing miR-206 and downregulating GREM1 in vivo

The xenograft model of CC was established in mice to research the role of circ_0007534 in vivo. As shown in Fig. 7a, b, the volume and weight of tumors were decreased in sh-circ_0007534 group in contrast to sh-NC group. The qRT-PCR showed that circ_0007534 and GREM1 levels were down-regulated but miR-206 expression was up-regulated in subcutaneous tumor tissues of sh-circ_0007534 group by comparison with sh-NC group (Fig. 7c). According to the protein images by western blot in Fig. 7d, we observed that the protein level of GREM1 was reduced in subcutaneous tumor samples with knockdown of circ_0007534. At least in part, knockdown of circ_0007534 suppressed tumor growth by regulating the miR-206/GREM1 axis in vivo.

**Fig. 7:** Inhibition of circ_0007534 reduced tumor growth partly by increasing miR-206 and downregulating GREM1 in vivo. (**a, b**) Knockdown of circ_0007534 reduced tumor volume (**a**) and weight (**b**) in mice. **c** The qRT-PCR was used to reveal the downregulation of circ_0007534, GREM1 and overexpression of miR-206 by silence of circ_0007534 in tumor tissues. **d** The protein level of GREM1 by western blot was decreased after circ_0007534 knockdown in tumor tissues. *NC* negative control, *GREM1* Gremlin1. All assays were performed for three times with technical n = 3. Statistical analysis was conducted by Student’s t-test and one-way analysis of variance followed by Tukey’s test. *P < 0.05, **P < 0.01

## Discussion

Exploring the molecular mechanism of CC progression is favorable for the therapeutic improvements for CC patients. The regulatory roles of circRNAs have been discovered in CC [28]. In the current report, knockdown of circ_0007534 was shown to impede the malignant behaviors of CC cells by the miR-206/GREM1 axis.

The dysregulated circRNAs can function as pro-cancer or anti-cancer factor in cancer progression. For instance, circ_0004507 was overexpressed in laryngeal cancer and it contributed to the malignance of cells [29]. Circ_0016760 was highly expressed in non-small cell lung cancer and enhanced cell proliferation, glycolysis [30]. Xie et al. found that circNR3C1 was downregulated and retarded the tumorigenesis of bladder cancer [31]. Li et al. affirmed the inhibitory effects of circ_0030998 on cell migration and invasion of lung cancer [32]. Circ_0007534 has been proved as an oncogenic circRNA in a handful of cancers. Due to the overexpression of circ_0007534 in CC tissues and cells, we used siRNA transfection to interference the circ_0007534 level for the functional research. Small interfering RNA (siRNA) is a common type of RNA interference (RNAi) that is intracellularly produced from exogenous synthetic oligonucleotides and can selectively knock down the expression of target in a sequence-specific way [33]. The function of circ_0007534 was then disclosed by analyzing the cellular processes after transfection of si-circ_0007534. Its expression knockdown inhibited cell viability, proliferation, invasion and promoted apoptosis in vitro.

The recent studies have paid attention on the sponge-like function of circRNAs for miRNAs. Hao et al. have identified that the regulation of circ_0007534 in pancreatic ductal adenocarcinoma was attributed to sponging miR-625 and miR-892b [34]. The sponge effects of circ_0007534 on miRNAs were also found in different cancers, such as miR-593 in breast cancer and miR-498 in CC [18, 35]. Differently, our results demonstrated that circ_0007534 was a sponge for miR-206. In addition, the oncogenic role of circ_0007534 in CC was partly achieved by inhibiting the expression of miR-206.

Some downstream targets for miR-206 have been reported in CC research, including BAG3 and G6PD [23, 24]. Moreover, Ji et al. also discovered that miR-206 suppressed the progression of CC by downregulating the expression of YWHAZ [36]. Chen et al. unraveled that miR-206 worked as a tumor inhibitor in CC by targeting Bcl-2 to regulate the hepatocyte growth factor (HGF)/c-Met pathway [37]. Our study validated that miR-206 targeted GREM1 in CC cells and the tumor-repressive role of miR-206 was achieved by targeting GREM1. Furthermore, we found that circ_0007534 increased the GREM1 level by sponging miR-206 and GREM1 overexpression rescued the si-circ_0007534-induced cancer inhibition in CC cells. Thus, the function of circ_0007534 might be associated with the miR-206-mediated expression upregulation of oncogenic GREM1.

GREM1 functions as a carcinogenic gene in variety of cancers and it is correlated to the activation of some signal pathway. For example, GREM1 is involved in the tumor promotion of breast cancer by activating the Akt/STAT3 signaling pathway [38]. Fu et al. declared that GREM1 activated the BMP signaling pathway in glioma to upregulate the expression of BMP2 and BMP4 proteins in the downstream [39]. GREM1 was also reported to activate the TGF-β/smad pathway to regulate proliferation, apoptosis, migration and invasion [40]. The effect of circ_0007534 on the development of CC might also be related to the GREM1-mediated signaling pathways.

Given the circ_0007534/miR-206 or circ_0007534/GREM1 network in regulating CC progression and the regulation of circ_0007534 on GREM1 expression by targeting miR-206, we considered that circ_0007534/miR-206/GREM1 axis was a novel molecular mechanism in the malignant progression of CC. Animal assay further confirmed that this signal axis was implicated in the tumor growth of CC in vivo. Thus, the circ_0007534/miR-206/GREM1 axis could be used for the target therapy for CC. RNAi technology provides an alternative of silencing specific target genes to control tumor growth [41]. Nanoparticles can act as the delivery vehicles to eliminate the rapid degradation and poor internalization of siRNA in vivo [41, 42]. Through combining with nanotechnology, siRNA of circ_0007534 can be delivered to the organism to inhibit the oncogenic GREM1 expression by acting on the miR-206/GREM1 axis. The malignant progression of CC may be repressed and the treatment can be improved.

The current study has certain limitations. Firstly, the larger numbers of clinical samples are needed to explore whether the dysregulation of circ_0000376 is related to the overall survival rate and survival time. Secondly, the downstream signalling pathways of GREM1 remain to be investigated. Additionally, it is interesting to analyze whether circ_0007534 can activate the signaling pathway via regulating the miR-206/GREM1 axis, which may provide a better understanding for how circ_0007534 acts in CC progression.

## Conclusion

In summary, our results clarified that circ_0007534 served as a sponge of miR-206 to upregulate the GREM1 expression to promote CC progression in vitro and CC tumorigenesis in vivo (Fig. 8). The miR-206/GREM1 axis is a different molecular mechanism for circ_0007534 in CC development, and the circ_0007534/miR-206/GREM1 signal network may lay the great foundation for circRNA research in the pathomechanism of CC.

**Fig. 8:** Circ_0007534/miR-206/GREM1 axis is involved in the regulation of CC cellular behaviors in vitro and tumor growth in vivo*. GREM1* Gremlin1

## Supplementary information

**Additional file 1: Figure S1.** Knockdown of circ_0007534 induced the proliferation inhibition in CC cells. BrdU assay revealed that cell proliferation was repressed after silence of circ_0007534. NC: negative control, DAPI: diamidine phenyl indoles. All assays were performed for three times with technical n = 3. Statistical analysis was conducted by Student’s t-test. *P < 0.05.

## Data Availability

The analyzed data sets generated during the present study are available from the corresponding author on reasonable request.
